The article "IoT Smart Agriculture and Agricultural Product Income Insurance Participant Behavior Based on Fuzzy Neural Network" was published in 2022. Journal: Comput Intell Neurosci.

# IoT Smart Agriculture and Agricultural Product Income Insurance Participant Behavior Based on Fuzzy Neural Network

**DOI:** 10.1155/2022/4778975

**Published:** 2022-05-29

**Authors:** Jiajia Tian, Dan Li, Xiaochen Jia

**Affiliations:** College of Economics and Management, Northeast Agricultural University, Harbin 150030, China

## Abstract

With the continuous development of modern science, more and more attention is paid to the application of science and technology for agricultural production. First of all, this article analyzes the development trend of modern agriculture, and designs the system through an overall plan of four parts: automatic acquisition, terminal control, network transmission, and cloud platform and terminal application. Taking automatic irrigation system and temperature automatic control system as examples, design an automatic control algorithm based on fuzzy neural network, and obtain the best control strategy through fuzzy inference and neural network training. Then, this paper studies the reliability of “price setting” in agricultural income insurance. This article takes the main crops of a certain province as an example to verify and analyze the risks of farmers' income levels from the viewpoint of corn yield risks and price risks, and advocate the necessity and feasibility of agricultural income insurance. Finally, from the perspective of different participants, this article analyzes the impact of insurance premium subsidies on the enthusiasm of agricultural producers to participate in insurance, the impact of insurance companies on the improvement of insurance operation efficiency in the planting industry, and the stability of the government's promotion of agricultural production. It also influences to design a set of IoT automatic control system for intelligent agriculture. The system realizes the acquisition and remote control of agricultural data by establishing an Internet of Things cloud platform, and uses automatic control algorithms based on fuzzy neural networks to realize automatic water-saving irrigation, automatic temperature control, and other functions. Based on this research, the main actions of joining agricultural income insurance and the participation model based on the perspective of tripartite participants.

## 1. Introduction

With the rapid development of economy and science and technology, the safety of food supply and sanitation has attracted more and more attention, which has led to an increasing demand for modern intelligent agricultural control systems with high accuracy and automation [1]. It is very important to establish the latest intelligent agricultural control system with high accuracy and automation. Since agriculture has various object characteristics, and the geographical environment is not fixed and the scope is relatively wide, the collection of agricultural data is full of challenges [2]. With the rapid development of Internet of Things (IoT) technology, its application prospects in agricultural systems are broad [3]. However, it is difficult for agricultural automatic control technology to correctly model environmental objects, and environmental data can be easily changed [4]. In this case, conventional PID control or neural network control of single fuzzy control cannot meet the requirements. The algorithm combining fuzzy control and neural network control can solve the above problems, which has a huge application value [5].

The article "IoT Smart Agriculture and Agricultural Product Income Insurance Participant Behavior Based on Fuzzy Neural Network" was published in 2022. Journal: Comput Intell Neurosci.

This theme aims to design a set of Internet automatic control system for intelligent agriculture. The system realizes functions such as automatic temperature control by establishing an IoT cloud platform [6]. At present, the development of agricultural income insurance is in the initial stage of pilot operation, and price setting is the core of the design of income insurance products [7]. The determination of the interest rate is based on the calculation of the long-term average loss rate that the farmer must pay the insurance premium to the insurance unit each year. Therefore, on the basis of this research, corn in a certain province, such as the price setting of agricultural income insurance, provides a reference standard for measuring the premium income of corn insurance in the province, and supports the reasonable design of agricultural income insurance, and other equivalent crop prices provide support. In addition, although planting insurance is gradually improving in China, there are also problems that cannot be ignored, such as a single subsidy method, few types of subsidy, high insurance premium rate, and guarantee level [8]. While increasing the scope of subsidies and increasing the amount of subsidies, the problems of planting insurance have not been effectively alleviated. This indicates that the establishment of a crop insurance performance evaluation system is the bottleneck of current agricultural development [9]. Therefore, this article is mainly based on agricultural production group insurance companies, governments. From the tripartite point of view of the participants in the performance evaluation, it is proposed to conduct a comprehensive analysis of the current insurance premium subsidy system, thereby constructing a performance evaluation system, and putting forward feasible suggestions for improving the insurance subsidy policy system of the planting industry, and helping to increase the use of insurance subsidies effectiveness [10].

The article "IoT Smart Agriculture and Agricultural Product Income Insurance Participant Behavior Based on Fuzzy Neural Network" was published in 2022. Journal: Comput Intell Neurosci.

## 2. Related Work

The literature puts the actions of farmers, government, and market on an equal and unified theoretical framework, analyzes the boundaries, functions, and roles of agricultural natural disaster risk management objects, understands how agricultural natural disaster risk management is carried out, and determines the risks at the same time and also the actions and factors influencing the decision-making actions of test subjects [11]. In order to analyze the risk of changes in the income of corn farmers, investigate and study the price of agricultural income insurance, and use the development experience of foreign agricultural income insurance to provide suggestions for improving the establishment of agricultural income insurance mechanisms in China [12]. The literature designed a crop monitoring system that uses visual technology to analyze the growth status of plants and realize real-time monitoring and online analysis plans [13]. The literature analyzes the behavior of farmers in purchasing agricultural insurance, and finally, from the perspective of adjusting the risks and relationships between the test subjects, it puts forward countermeasures and suggestions to promote the sustainable and stable development of agricultural insurance [14]. Documents based on the theory of complex adaptability (CAS) analyzed the complexity of the agricultural product “price insurance + futures” model and the application mechanism of the agricultural “price insurance + futures” system [15]. At the same time, a complex adaptation system (CAS) is used to establish a monitoring system and a risk management system for the rising prices of agricultural products. The literature is based on the background of intelligent agriculture, combined with the experience of urban modern agricultural incorporation courses, and discusses the educational reform of the incorporation courses in agricultural and forestry universities [16]. The literature studied the practical problems in intelligent agricultural production and management, in order to realize the functions of data collection, management, and control [17].

## 3. IoT Smart Agriculture Design Based on Embedded Processor

### 3.1. The Overall Scheme Design of the System

The block diagram of the IoT automatic control system for smart agriculture designed in this subject is shown in Figure 1.

The automatic acquisition/control terminal can realize the signal input and output in the agricultural field. Considering that there are many types of acquisition and control in the agricultural field, the system uses a high-performance embedded processor based on ARM equipped with various sensors and controllers in order to complete the acquisition and control of information. The system sends the collected data to the cloud platform and can be sent to the form. The cloud platform runs on a core server, and the core server mainly receives collected information returned through the network. This system has designed the web page of the automatic control system of the Internet of Things for intelligent agriculture. Web pages can be accessed through mobile phones, smart TVs, and computers. Users can correctly grasp the situation of agricultural land through the pages, and operate on-site controllers through the pages.

The article "IoT Smart Agriculture and Agricultural Product Income Insurance Participant Behavior Based on Fuzzy Neural Network" was published in 2022. Journal: Comput Intell Neurosci.

### 3.2. Design of Agricultural Automatic Control Algorithm

In the active control mode of the automatic acquisition/control terminal, the fuzzy control system is composed of five main parts: the selection of input variables, fuzzification, fuzzy inference, fuzzy solution, and system output. The neural network analysis algorithm can learn the field data and obtain the best control strategy, but it cannot handle fuzzy information. In the agricultural field, not only can it handle vague information, but it can also obtain the best control rules through training.

The topological structure of the fuzzy neural network is shown in Figure 2.

The transmission rules between each 2 layers of the fuzzy neural network are as follows

(1) $$\begin{array}{c} {\text{net}}_{i}^{k}=w_{ij}^{k}\cdot u_{j}^{k}, \end{array}$$

where net; the input of the *k*-th layer node;

*w*_*ij*_^*k*^——the connection weight between the *i*-th node of the *k* layer and the *j* node of the *k* − 1 layer.

*u*_*j*_^*k*^——in the *j*-th input connected to the *i*-th node, *o*_*i*_^*k*^ represents the output of the *k*-layer node.

The relationship between the input and output of the first layer is as follows:

(2) $$\begin{array}{c} {\text{net}}_{i}^{k}=w_{ij}^{1}*u_{j}^{1},\\ o_{i}^{1}={\text{net}}_{i}^{1}. \end{array}$$

The second layer is the membership function layer. Input variables generally describe the membership relationship. The input and output relationships are as follows:

(3) $$\begin{array}{c} {\text{net}}_{i}^{2}=-\left(\frac{{\left(u_{j}^{2}-m_{ij}\right)}^{2}}{{\left(\sigma_{ij}\right)}^{2}}\right),\\ o_{i}^{2}=\exp\left({\text{net}}_{i}^{2}\right), \end{array}$$

where *m*_*ij*_- the average value of the *j*-th input relative to the *i*-th member function.

*σ*_*ij*_——the variance of the *j*-th input relative to the *i*-th member function;

*o*_*i*_^2^ 0; - the output of the second layer node.

The third layer is the control rule layer that deals with all the fuzzy control rules. The input and output relationship of the *i*-th rule is as follows:

(4) $$\begin{array}{c} {\text{net}}_{i}^{3}=\overset{n}{\underset{j=1}{∐}}w_{ij}^{3}u_{j}^{3},\\ o_{i}^{3}={\text{net}}_{i}^{3}. \end{array}$$

The fourth layer is the output layer, which outputs the data processed by the network. The input and output relationship of the *i*-th output unit of this layer is as follows:

(5) $$\begin{array}{c} {\text{net}}_{i}^{43}=\sum_{i=1}^{n}w_{ij}^{4}u_{j}^{4},\\ o_{i}^{4}={\text{net}}_{i}^{4}. \end{array}$$

Before training the neural network, the objective function is as follows:

(6) $$\begin{array}{c} E=\frac{1}{2}\sum_{i}{\left(d_{i}^{4}-o_{i}^{4}\right)}^{2}\\ =\frac{1}{2}\sum_{i}{\left(d_{i}^{4}-f^{4}\left({\text{net}}_{i}^{4}\right)\right)}^{2}. \end{array}$$

After neural network training, when the system is running in automatic control mode, it can realize automatic control according to the set control rules.

The article "IoT Smart Agriculture and Agricultural Product Income Insurance Participant Behavior Based on Fuzzy Neural Network" was published in 2022. Journal: Comput Intell Neurosci.

### 3.3. System Hardware Design

The camera uses STM32 to control the camera to take photos and obtain the original image of the complete set of equipment. The main parameters are shown in Table 1.

The MG811 solid electrolyte sensor is put into the detection gas and the following electrochemical reaction occurs:

Positive electrode:

(7) $$\begin{array}{c} 2N_{a}^{+}\frac{1}{2}O_{2}+2e^{-}=N_{a_{2}}O. \end{array}$$

Negative electrode:

(8) $$\begin{array}{c} 2L_{i}^{+}+CO_{2}+\frac{1}{2}O_{2}+2e^{-}=L_{i_{2}}CO_{2}. \end{array}$$

### 3.4. System Software Design

The control system of this theme includes multiple data collection expansion boards consisting of core control boards, substations, PC control terminals, and a single Internet cloud platform. Build a cloud platform to realize the communication mechanism between the control system and the cloud platform, as well as the communication mechanism between the control board and the external data collection board. In the passive control mode, the best control rules are obtained through fuzzy modeling and network training. At the same time, when the field sensor data is abnormal or the field actuator fails, the core controller will actively send out an alarm and report the error information to the cloud platform. The flowchart of the system software is shown as in Figure 3.

The control board executes the UCOS-II operating system. After initialization, it mainly performs six tasks: maintain MODBUS register table software design, acquisition of analog input data, acquisition of digital input data, control of digital output, 3G communication with the cloud platform, and configuration of the control board.

#### 3.4.1. Maintain MODBUS Register Table Software Design

The control card allocates 300 registers to each expansion board to store the information of the expansion board, and the corresponding register that controls the data of the Modbus register of the expansion board. When the control board sends a control command to the expansion board, the control board will change the corresponding register value in the expansion board and send the control information through the mail box. After the expansion board receives the control information, it will control the corresponding output level. In the communication between the control panel card and the cloud platform, output control tasks are performed through the message mailbox.

The article "IoT Smart Agriculture and Agricultural Product Income Insurance Participant Behavior Based on Fuzzy Neural Network" was published in 2022. Journal: Comput Intell Neurosci.

Modubus protocol is a bus protocol suitable for applications in the agricultural field. Through the Modubus protocol, the first set of registers stores the information of the control board, and the second set of registers stores the information of 9 expandable data collection expansion boards.

#### 3.4.2. Design of Analog Data Acquisition Software

In this task, when the board is operating in passive control mode, the automatic control algorithm is not executed. When the board is running in the automatic control mode, it will execute the automatic control algorithm based on fuzzy neural network to control the digital switch.

#### 3.4.3. Digital Data Acquisition Software Design

In this task, the sampled data is written into the corresponding register through level conversion. Next, determine whether the digital quantity has changed. When the digital quantity changes, the signal needs to be sent to the 3G communication task for prompting.

#### 3.4.4. Digital Output Control Software Design

In the digital output task, after receiving the signal, the corresponding digital channel switch will be set.

#### 3.4.5. 3G Communication Software Design

In this task, the data collected by the main control board is sent to the cloud platform via a short connection every 5 seconds.

#### 3.4.6. Configuration Control Board Software Design

In this task, the user can change the control board information through the serial port. At the same time, in the information composition process, after unlocking the control board chip FLASH, the composition information stored in the FLASH must be changed through the serial port. If the flash information is locked, the composition information of the layout card will be changed.

### 3.5. Internet of Things Cloud Platform Construction

On the cloud platform, web pages are made based on the Bootstrap framework. Web pages can be constructed according to the specific conditions of each monitoring system. Digital data and analog data are displayed in the form of charts and graphs on the page, so the monitor can intuitively and accurately understand the status of the website.

The article "IoT Smart Agriculture and Agricultural Product Income Insurance Participant Behavior Based on Fuzzy Neural Network" was published in 2022. Journal: Comput Intell Neurosci.

### 3.6. System Function Test

The automatic control algorithm function designed by this project is tested by the irrigated farmland and greenhouse sampling data of the China Agricultural Information Database. The system runs in active control mode, and the soil moisture potential target is set to 0 (soil moisture is appropriate). As shown in Table 2:

As can be seen from the above table, in the modeling process, factors such as temperature and lighting are not considered. If the lighting is excessive or evaporates, the actual irrigation time may be slightly longer than the output time of the automatic irrigation system. In summary, the automatic irrigation control system designed in this paper can meet the requirements of the agricultural automatic control.

In the automatic temperature control system test, 2000 sets of temperature difference, temperature change rate, and ventilation time data are used as training samples for neural network algorithms. The training sample data is trained by MATLAB software to obtain optimized membership functions and fuzzy control rules. The software program is created to control the opening and closing time of the ventilation valve.

The system operates in the activity control mode, setting a temperature target of 25°C in a non-heated, ventilated sightseeing greenhouse. This solar greenhouse maximizes the use of solar energy, and maintains the temperature required for crop growth through the storage and release of heat in the greenhouse. The data of 20 sets of verification samples are selected and input into the system. As shown in Table 3, according to the member function after training, the output result is compared with the field data to verify the automatic temperature control system.

It can be seen from the table that in an agricultural field, if the temperature rises too fast, the actual ventilation time may be slightly longer than the output time of the automatic temperature control system. In general, the temperature automatic control system designed by this theme can meet the requirements of agricultural automatic control.

The functions of the control panel card and the cloud platform are tested using the data from the breeding monitoring substation of the Chinese Academy of Agricultural Sciences. The dissolved oxygen, pH value, and water temperature data collected by the analog input channel will be displayed on the web page. According to the state of the switch, the switching status of the solenoid valve, the peristaltic pump, and the recovery pump will be displayed. The test results show that the DeviceHive IoT cloud platform can correctly receive and save the simulated data sent from the control board, and realize the monitoring and control of agricultural data through the web.

The article "IoT Smart Agriculture and Agricultural Product Income Insurance Participant Behavior Based on Fuzzy Neural Network" was published in 2022. Journal: Comput Intell Neurosci.

## 4. Research and Analysis on the Behavior of Participants in Agricultural Income Insurance

### 4.1. The Concept of Agricultural Income Insurance

#### 4.1.1. Agricultural Income Risk

From the perspective of agricultural income insurance, this article advocates the concept of agricultural income risk. The concept of agricultural income risk can be defined as the sum of irresistible and resistible risks that affect the farmers' income after planting. Specifically, it includes climate factors, natural factors, market factors, policy factors, and the risk of farmers losing the income of agricultural operators. In fact, the agricultural income risk of farmers mainly covers the risk of output during the production process and the risk of market price fluctuations. But it is not limited to this. All risks that affect farmers' agricultural production and operating income loss can be called agricultural risks.

#### 4.1.2. Agricultural Product Income Insurance

Agricultural income insurance means that if the insurance contract covers the reasons for the agricultural harvest, the expected income level is lower than the level of certain safety, and the insurance contractor within the insurance liability covers the agricultural income level with the theme of planting crop products, and agricultural income insurance underwrites. People agree to pay the difference between the level of income protection and actual income.

### 4.2. Determination Method of Agricultural Income Insurance Premium

Since the income fee set in the first step is filtered, this paper analyzes the income risk mechanism of corn farmers in a certain province that has been filtered by the HP corn production and price series. This chapter continues to filter the processed data. Because the *β* of the independent variable value is distributed in the range of [0, 1], this chapter first performs the filtering process for the data to be normalized, and all the independent variable values are configured in the interval [0, 1]. After processing corn production and price data, this chapter first creates descriptive statistics for the selected data, and displays the statistical results in Table 4.

Second, the Jarque–Bera method and the Kolmogorov–Smirnov method were used to test the regularity of the corn production and price series in a certain province. The JB test statistic of maize yield sequence is 5.7579, and the *P* value is 0.0561. The KS statistics is 0.31, and the *P* value is 7.4235.10. The JB test statistic of the price series of corn is 14.4178, and the *P* value is 0.0074. The KS statistics is 0.20, and the *P* value is 9.3241 E-20°. The test results are shown in Table 5. From the *P* value results of the JB test and the KS test, it can be seen that the yield and price series of corn are not suitable for the normal distribution, so this paper chooses other distributions for implementation and performs distributed fitting to the selected data.

The article "IoT Smart Agriculture and Agricultural Product Income Insurance Participant Behavior Based on Fuzzy Neural Network" was published in 2022. Journal: Comput Intell Neurosci.

According to the statistics of this paper, it is found that the output and price series of corn in a certain province are not suitable for normal distribution. In view of this, this paper selects a distribution with a good fitting effect based on the results of previous literature research. In the second chapter of this article, in the previous research on fitting the marginal distribution, it was found that the lognormal distribution is mostly the best fitting effect of typical agricultural production data. Logical distribution and gamma distribution are the most representative and best distributions of agricultural price data series. Based on the differences in agricultural development and agricultural product price determination mechanisms at home and abroad, this article will focus on the selection type of the peripheral distribution of domestic insurance prices, and finally select the “EZTW” distribution, lognormal distribution, and other distributions for maize output data per unit area distribution fitting.

The probability density function and parameter range of the yield sequence are as follows:

(1) Weibull distribution density function:
  (9) $$\begin{array}{c} f\left(x\right)=\frac{\alpha }{\beta }{\left(\frac{x}{\beta }\right)}^{\alpha -1}\exp\left(-{\left(\frac{x}{\beta }\right)}^{\alpha }\right),\;x\geq 0. \end{array}$$
(2) Lognormal distribution probability density function:
  (10) $$\begin{array}{c} f\left(x\right)=\frac{1}{x\sqrt{2\pi }\sigma }e^{{\left[\ln\left(x\right)-\mu \right]}^{2}/2\sigma^{2}},\;x\geq 0. \end{array}$$
(3) Beta distribution probability density function:
  (11) $$\begin{array}{c} f\left(x\right)=\frac{1}{b\left(a_{1},a_{2}\right)}\frac{{\left(x-a\right)}^{a_{1}-1}{\left(b-x\right)}^{a_{2}-1}}{{\left(b-a\right)}^{a_{1}+a_{2}-1}},\;a\leq x\leq b. \end{array}$$
The probability density function and parameter range of the price series are as follows:
(4) Logistics distribution probability density function:
  (12) $$\begin{array}{c} f\left(x\right)=\frac{e^{-\left(x-\mu \right)/\sigma }}{\sigma {\left(1+e^{-\left(x-\mu \right)/\sigma }\right)}^{2}},\;-\infty <x<+\infty . \end{array}$$
(5) Burr distribution probability density function:
  (13) $$\begin{array}{c} f\left(x\right)=\frac{ak{\left(x/\beta \right)}^{\alpha -1}}{\beta {\left(1+{\left(x/\beta \right)}^{\alpha }\right)}^{k+1}}\;x\geq 0. \end{array}$$
(6) Gamma distribution probability density function:

(14) $$\begin{array}{c} f\left(x\right)=\frac{\beta^{\alpha }x^{\alpha -1}e^{-x\beta }}{\Gamma \left(\alpha \right)},\;x\geq 0. \end{array}$$

The article "IoT Smart Agriculture and Agricultural Product Income Insurance Participant Behavior Based on Fuzzy Neural Network" was published in 2022. Journal: Comput Intell Neurosci.

#### 4.2.1. Distribution Fitting Results

In this paper, lognormal distribution and *β* distribution are selected, and the distribution fitting of maize yield data per unit area is carried out. In order to match the price series of corn, logical and gamma distributions were chosen. The fitting distribution based on the KS test is good. The smaller the KS test value, the better the distribution fitting effect. This article classifies the advantages of the adaptability test, and finally concludes that the Weibull distribution is the most suitable for a certain province's maize yield sequence per unit area, and the *β* distribution is the most suitable for the maize price sequence, as shown in Table 6.

It can be seen from Table 6 that the tolerance distribution KS test value of the unit area corn yield series is 0.0979, which is lower than the 0.165 and 0.0982 of the fitted statistics of the *β* distribution and the lognormal distribution. Therefore, the fitting effect of the expandable distribution of the maize yield series per unit area is very good. Therefore, the probability density function of the price distribution of corn production is as follows:

(15) $$\begin{array}{c} f\left(x\right)=0.017\times {\left(\frac{x}{52}\right)}^{-0.12}\exp^{-{\left(x/52\right)}^{0.88}}. \end{array}$$

The fitting results of maize yield sequence are shown in Figure 4:

The results of the goodness of fit test of the corn price series distribution are shown in Table 7.

As shown in Table 7, the KS test statistics of the Burr distribution of the corn price series is 0.19, the Logistics test value is 0.184, and the Gemmak's test value is 0.1672. The statistic of Burks test is the smallest, so it is the best approximate distribution. Therefore, this paper selects the distribution and constructs the subsequent simultaneous distribution function by fitting the price series of corn. The parameters *α* is 0.7106, *β* is 32, and *k* is 0.4293. The probability density function of the corn price distribution is as follows.

(16) $$\begin{array}{c} f\left(x\right)=\frac{0.3\times {\left(x/32\right)}^{-0.31}}{32\times {\left(1+{\left(x/32\right)}^{0.71}\right)}^{1.43}}. \end{array}$$

The results of corn price series distribution fitting are shown in Figure 5:

#### 4.2.2. Choice of Copula Function

After obtaining the best-fitting distribution of corn yield and price, the multivariate Copula function is used to calculate the correlation between yield and price, and a simultaneous distribution function can be constructed. In this article, in order to estimate the joint distribution of corn yield and price in a certain province, a two-stage maximum likelihood estimation method is used to select the best type of Copula function from the least squares Euclidean distance. The specific calculation results are shown in Table 8.

The article "IoT Smart Agriculture and Agricultural Product Income Insurance Participant Behavior Based on Fuzzy Neural Network" was published in 2022. Journal: Comput Intell Neurosci.

This chapter uses the least squares Euclidean distance method to estimate various Copula functions. It can be seen that there is a slight positive correlation between corn production and price in a certain province. Therefore, the Gumbel Copula function parameter 1.0000 is selected as the initial parameter of the data simulation, and the corresponding inverse function value is calculated according to the marginal distribution function of the yield and price, and the corn income is estimated.

### 4.3. Analysis of Participation Behavior Based on the Perspective of Three Participants

#### 4.3.1. Analysis of the Effect of Premium Subsidies on the Improvement of the Enthusiasm of Agricultural Production Entities

This chapter uses a binary response model to analyze the influencing factors of the willingness of agricultural production entities to pursue insurance. The specific form of the model is the logit model:

(17) $$\begin{array}{c} P\left(y=1|x\right)=F\left(x,\beta \right)\\ =\Lambda \left(x^{\prime }\beta \right)\\ =\frac{x^{\prime }\beta }{1+\exp\left(x^{\prime }\beta \right)}. \end{array}$$

In the formula, *Y* is a binary selection variable, indicating whether the agricultural production object continues to increase planting insurance. *P*(*y* = 1) is the probability of *y* = 1. The value of *β* can be calculated using the most likelihood inference algorithm. The following formula can be used to estimate the limiting effect of the *i*-th explanatory variable:

(18) $$\begin{array}{c} mfx_{i}=\frac{\partial P\left(x\right)}{\partial x_{i}}\\ =g\left(x^{\prime }\beta \right)\beta_{i}. \end{array}$$

In the formula, *mfx* shows that the change of variables has an impact on the probability of agricultural production entities continuing to increase planting insurance. *G*(^*∗*^) is the probability density function.

This chapter uses the Logit model to analyze the impact of planting insurance subsidies on the insurance intentions of agricultural producers. The verification results are shown in Table 9.

The results show that with the increase of insurance subsidies, the insurance enthusiasm of agricultural producers has greatly increased, and other factors have also affected the insurance enthusiasm of agricultural producers from different perspectives.

*(1) The Impact of Premium Subsidies*. The results of the model show that the intensity of premium subsidies has a great impact on the enthusiasm of agricultural producers to promote insurance. For every additional 100 units of subsidies, agricultural producers' enthusiasm for insurance increases by 0.43 percentage points. This is because with the increase in insurance premium subsidies, agricultural producers can make their incomes more stable.

*(2) The Impact of Agricultural Income*. Agricultural income has a great influence on increasing the enthusiasm of agricultural producers to invest in insurance. Whenever agricultural income increases, the enthusiasm of agricultural producers for insurance increases by a rate of 0.002. This shows that the higher the agricultural income, the higher the demand of agricultural producers in order to avoid the risks of agricultural operations, and the correspondingly higher the enthusiasm for purchasing planting insurance.

*(3) The Influence of Education Level*. The level of education has a great influence on increasing the enthusiasm of agricultural producers for insurance investment. The enthusiasm of agricultural producers for insurance increased by 0.226 percentage points with the improvement of education level. This shows that the higher the education level of agricultural producers, the higher their awareness of planting insurance and agricultural business risks, and the higher their willingness to purchase planting insurance.

*(4) Other Insignificant Variables*. The results of the model show that the area of arable land, the existence of family village cadres, and the total family income have a positive effect on agricultural producers' insurance, while the ratio of grain area and the intention to promote insurance has a mutually inhibiting relationship. The larger the area of arable land, the higher the possibility of agricultural producers facing operational risks and the stronger the tendency to purchase planting insurance. On the other hand, the increase in planting insurance premiums may lead to a decline in the willingness of agricultural producers to purchase planting insurance, but the impact is not significant. Village cadres play a leading and exemplary role in agricultural production and operation, and are better able to understand insurance contracts and planting industry information than ordinary peasant families. The total household income includes agricultural income and non-agricultural income, which are affected by many factors, but have no great influence on the willingness to upgrade insurance. The higher the proportion of grain area, the lower the diversity of agricultural production objects, and the lower the willingness to buy planting insurance. Although it shows a negative relationship, the effect is not obvious.

The article "IoT Smart Agriculture and Agricultural Product Income Insurance Participant Behavior Based on Fuzzy Neural Network" was published in 2022. Journal: Comput Intell Neurosci.

#### 4.3.2. Analysis of the Effect of Premium Subsidies on the Efficiency Improvement of Insurance Company Plantation Insurance Operations

The DEA model is a model proposed by FAREL's production efficiency framework based on relative efficiency measurement. In order to measure the operational efficiency of an organization, the “input-output ratio” is usually used

(19) $$\begin{array}{c} E=\frac{\text{OUT}}{\text{IN}}. \end{array}$$

Here, *E* represents the operating efficiency of the organization, OUT represents output, and IN represents input.

The Malmquist index is based on the DEA method, which uses panel data to measure the productivity of all factors. It can explain the dynamic change of relative efficiency over a period of time. When the change of all factor productivity is greater than 1, the efficiency level will increase. The formula for Malmquist index is as follows:

(20) $$\begin{array}{c} \text{tfp}={\text{tec}}^{*}\text{efc}\\ ={\text{tec}}^{*}\left({\text{pech}}^{*}\text{sech}\right). \end{array}$$

Here, TTP represents the changes in the production of all factors, and can be decomposed into technological progress (TEC) and comprehensive technological efficiency changes (EFC).

In this chapter, in order to analyze the operational efficiency of the plantation insurance business of the five insurance companies in *J* City, the technical efficiency of the plantation insurance business of the insurance company is decomposed into pure technical efficiency and scale efficiency. The estimated results of the model are shown in Table 10.

It can be seen from Table 10 that in 2013, the companies with the highest pure technical efficiency (1.000) in the plantation insurance business were China Life Insurance, China Insurance, and PICC. The pure technical efficiency of the five companies in 2017 and 2018 was all 1.

#### 4.3.3. Analysis of the Effect of Premium Subsidies on the Government's Promotion of Agricultural Production Stability

The Cobb Douglas production function is one of the classic functional models for analyzing the industrial relations of industrial sectors. The basic form is as follows:

(21) $$\begin{array}{c} Y=AL^{\alpha }K^{\beta }\;u. \end{array}$$

Take the logarithm to get

(22) $$\begin{array}{c} \ln\left(Y\right)=\ln\left(A\right)+\alpha \;\ln\left(L\right)+\beta \;\ln\left(K\right). \end{array}$$

Because it is difficult to quantify the stability of the agricultural production, this chapter will use the total agricultural output value to determine the stability of agricultural production and investigate the impact of insurance premium subsidies and other agricultural inputs on the total agricultural output value.

The article "IoT Smart Agriculture and Agricultural Product Income Insurance Participant Behavior Based on Fuzzy Neural Network" was published in 2022. Journal: Comput Intell Neurosci.

According to the model constructed with the Cobb Douglas production function, the parameter estimation results obtained by the regression method are shown in Table 11. The input and output elasticity is 1.5%, but the output elasticity is not obvious. However, judging from the crossover period of insurance premium subsidies after 2012, the elasticity of insurance premium subsidies has increased by 0.8%. After 2012, with the increase in insurance subsidies for planting industries, insurance premium subsidies are used in agricultural production. They play an increasingly important role in its stability.

From the point of view of the elasticity of other factors, the industry correlation elasticity of insurance premium income of the planting industry is 5.1%, which is meaningful at the level of 5%. Since 2012, the insurance premium income elasticity of plantation insurance has increased by 2.7 percentage points. With the development of plantation insurance, plantation insurance has played a significant role in promoting agricultural production and improving the value of agricultural output. The industrial correlation elasticity of rural labor to the total agricultural output value is 14.6%, which is meaningful at the 1% level. The input and output elasticity of agricultural production value to the total output of agricultural machinery is 32.2%, but its impact is not significant from the perspective of effectiveness.

## 5. Conclusion

It can be seen from the analysis results of this article that under the same guarantee level, the insurance cost of agricultural income insurance will be lower than the insurance cost of other combination products of the same guarantee level. Under the same payment, income insurance for agricultural products has a higher level of guarantee. This undoubtedly reflects the efficient characteristics of agricultural income insurance. The income of agricultural products is still in the experimental stage and needs long-term implementation and development, so it is necessary to use research and other supporting policies. Under the same financial and agricultural subsidies, agricultural income insurance has a high degree of guarantee, which helps to improve the overall social benefits. Regarding the financial subsidies of local governments, the central government clearly defines the importance of agricultural support. According to the actual conditions of each region, it is obliged to provide planned subsidies to the local agricultural economy to reduce the burden on farmers.

The survey of planting insurance premium subsidies from the perspective of the tripartite main bodies of agriculture shows that increasing planting insurance premium subsidies will increase the enthusiasm of agricultural producers. The increase in insurance premium subsidies has a great impact on the enthusiasm of agricultural production entities to purchase insurance. Through static operating efficiency analysis, the overall operating efficiency of the planting insurance business of the five insurance companies has been improving. However, the efficiency of agricultural insurance companies' plantation insurance scale is generally lower than that of pure technology. Through the analysis of dynamic utilization efficiency, it can be concluded that the overall production efficiency of plantation insurance of all agricultural insurance companies in *J* City shows a reverse “*U*”-shaped tendency. Although the impact of premium subsidies on total agricultural production is relatively limited, after 2012, with the increase in insurance subsidies for the planting industry, premium subsidies have played an increasingly important role in stabilizing total agricultural production.

The article "IoT Smart Agriculture and Agricultural Product Income Insurance Participant Behavior Based on Fuzzy Neural Network" was published in 2022. Journal: Comput Intell Neurosci.

## Figures and Tables

**Figure 1:** Block diagram of agricultural automatic control system.

**Figure 2:** Fuzzy neural network topology.

**Figure 3:** System software flowchart.

**Figure 4:** Sequence fitting distribution of maize yield.

**Figure 5:** Fitting distribution of corn price series.

**Table 1:** Camera parameters.

Parameter	Parameter value
I/O voltage	2.5–3.0 V
Power consumption	60 mW/15 fps
Optical size	1/6 inch
Sensitivity	1.3 v/(Lux-sec)
Signal-to-noise ratio	46 dB
Photosensitive array	640 × 480

**Table 2:** Automatic irrigation system output and field data comparison result.

Serial number	Soil water potential	Rainfall	Field data	Irrigation system output	Serial number	Soil water potential	Rainfall	Field data	Irrigation system output
1	M	S	LS	VS	11	RL	S	L	L
2	RM	S	LS	LS	12	RL	M	M	M
3	RM	L	LS	LS	13	RM	L	VS	VS
4	RL	S	L	L	14	M	L	VS	VS
5	M	VL	VS	VS	15	RL	M	M	M
6	M	S	VS	VS	16	RL	VL	VS	VS
7	RL	S	VL	L	17	VL	S	VL	VL
8	RL	S	L	L	18	RM	L	VS	VS
9	RM	M	VS	VS	19	RM	S	M	LS
10	VL	S	VL	VL	20	M	S	VS	VS

**Table 3:** Comparison result of temperature automatic control system output and field data.

Serial number	Temperature change rate	Temperature difference	Field data	Temperature control system output	Serial number	Temperature change rate	Temperature difference	Field data	Temperature control system output
1	N	PS	S	S	11	Z	PS	S	S
2	Z	PM	L	L	12	N	N	S	S
3	N	N	S	S	13	PS	PM	VL	L
4	N	Z	S	S	14	Z	PM	L	L
5	PS	Z	S	S	15	PB	PM	VL	VL
6	PS	PS	M	M	16	Z	PM	L	L
7	PM	PM	VL	L	17	N	Z	S	S
8	Z	PM	L	L	18	N	PS	S	S
9	PM	PB	VL	VL	19	PS	PS	M	M
10	PS	Z	S	S	20	PS	Z	S	S

The article "IoT Smart Agriculture and Agricultural Product Income Insurance Participant Behavior Based on Fuzzy Neural Network" was published in 2022. Journal: Comput Intell Neurosci.

**Table 4:** Descriptive statistical analysis of maize yield and price series.

	Mean	Standard deviation	Skewness	Kurtosis

Yield	8.3516	0.2116	−0.8952	3.4996
Price	106.2574	9.7605	1.0877	4.9793

**Table 5:** Analysis on normality test of maize yield and price series.

	JB inspection		KS inspection		Test result
	JB statistics	*P* value	KS statistics	*P* value	

Yield	5.7578	0.0563	0.32	7.4235*e* − 10	Non-normal distribution
Price	14.4177	0.0072	0.20	9.3241*e* − 20	Non-normal distribution

**Table 6:** Test on the goodness of fitting distribution of maize yield series.

Fitted distribution type	KS test statistics	Sort
Weibull	0.0978	1
Beta	0.1164	3
Lognormal	0.0983	2

**Table 7:** Test on the goodness of fitting distribution of maize price series.

Fitted distribution type	KS test statistics	Sort
Burr	0.1093	1
Logistic	0.1385	2
Gamma	0.1673	3

**Table 8:** Multiple copula function maximum likelihood method estimation results.

Function type	Parameter	Rank correlation coefficient	Least square euclidean distance
Normal Copula	−0.0422	−0.0267	0.0365
*t*-Copula	−0.0413	−0.0265	0.0364
Frank Copula	−0.2072	−0.0230	0.0362
Gumbel Copula	1.0000	1.3575*e* − 06	0.0328
Clayton Copula	1.4509*e* − 06	7.2543*e* − 07	0.0327

**Table 9:** Logit model analysis results of agricultural production entities' willingness to purchase insurance.

Variable	Unit	Marginal effect	Standard deviation
Intensity of premium subsidies	Hundred yuan	0.430^*∗∗∗*^	0.026
Cultivated area	mu	0.003	0.005
Proportion of grain area	%	−0.532	1.126
Is there a village cadre at home	1 = Yes, 0 = No	0.412	0.588
Total household income	yuan	0.002	0.003
Agricultural income	yuan	0.003^*∗*^	0.002
Education level	year	0.227^*∗*^	0.124
Constant term	—	0.174	0.176
*R*-squared	—	0.169	

**Table 10:** The pure technical efficiency of the plantation insurance business of five insurance companies in *J* City, 2013–2018.

Years	Company abbreviation					
	China pacific insurance	China life insurance	China insurance	Anwar insurance	Chinese People's insurance	Mean
2013	0.892	1.000	1.000	0.973	1.000	0.973
2014	1.000	1.000	1.000	1.000	1.000	1.000
2015	1.000	1.000	1.000	1.000	1.000	1.000
2016	0.926	1.000	1.000	1.000	1.000	0.985
2017	1.000	1.000	1.000	1.000	1.000	1.000
2018	1.000	1.000	1.000	1.000	1.000	1.000

**Table 11:** *C*-*D* production function estimation result.

Variable	Coefficient	Standard deviation
Premium subsidy (logarithmic)	0.016	0.015
Premium income (logarithmic)	0.052^*∗∗*^	0.024
After 2012 × logarithm of premium subsidies	0.007^*∗*^	0.004
After 2012 × logarithm of premium income	0.026^*∗∗*^	0.012
Rural labor force (logarithm)	0.147^*∗∗∗*^	0.012
Total power of agricultural machinery (logarithm)	0.321	0.342
Actual cultivated land area at the end of the year (logarithm)	0.773^*∗*^	0.386
Contribution rate of technological progress	0.151^*∗∗∗*^	0.017
*R*-square	0.972	
Ptob > *F*	0.000	

The article "IoT Smart Agriculture and Agricultural Product Income Insurance Participant Behavior Based on Fuzzy Neural Network" was published in 2022. Journal: Comput Intell Neurosci.

## Data Availability

The data used to support the findings of this study are available from the corresponding author upon request.
